# Panax Notoginseng Saponin Rg1 Can Effectively Improve the Cognitive Function of 5 × FAD Mice

This article has been retracted.

**DOI:** 10.1155/2022/5152761

**Published:** 2022-04-11

**Authors:** Lili Guo, Kun Li, Jiajun Zhou, Lian Luo

**Affiliations:** Department of Neurology, Hangzhou Xixi Hospital Affiliated to Zhejiang University of Traditional Chinese Medicine, Hangzhou 310024, China

## Abstract

In order to investigate the effect of notoginsenoside Rg1 on cognitive function in 5*∗*FAD mice and the mechanism of Cx43 in improving cognitive function in mice, the methods 5*∗*FAD mice are selected as experimental animals and normal mice as healthy control. They were divided into three groups: healthy control group (*n* = 10), disease group (*n* = 10), and treatment group (*n* = 10, Panax notoginsenoside Rg 1150 mg/kg/d) for 2 months. Two months later, three groups of mice were subjected to classical water maze and Y-maze to test the cognitive ability of mice, and the correct response times and total response time were recorded. At the end of the cognitive function test, the mice were executed, and the brain tissues were taken. The expression of Cx43 protein and the changes of glial cells and neurons in the brain of the mice were analyzed at the cellular level. After treatment with Panax notoginseng saponin Rg 1150 mg/kg/d, it was found that the escape latency of mice in the treatment group was significantly lower than that in the disease group from the third day of training (*P* < 0.05); the time spent on the platform quadrant and the number of times crossing the platform in the treated mice were significantly increased, and the difference was statistically significant (*P* < 0.05); the expression of Cx43 protein in the brain of mice after treatment was significantly higher than that of mice in the disease group (*P* < 0.05). *Conclusion.* Panax notoginseng saponin Rg1 can effectively improve the cognitive function of 5*∗*FAD mice by increasing the secretion of Cx43 protein, thus increasing the reactivity of glial cells and neurons.

## 1. Introduction

With the advent of an aging society in China, China will become the country with the largest number of Alzheimer's disease (AD) patients [1, 2]. Previous studies have shown that the cortex and hippocampus of AD patients are the most damaged brain areas. Recent studies have shown that Panax notoginseng saponin Rg1 can increase the expression of connexin 43 (Cx 43) in the brain, thereby improving the related symptoms of AD patients [3], but its specific mechanism is still unclear. The aim of this study was to observe the effect of notoginsenoside Rg1 on cognitive ability in mice by using a 5xFAD mouse model and to explore the mechanism of Cx43 interaction between glia and neurons in mice, so as to provide the basis for screening possible clinical drug targets [4].

A randomized controlled study was designed. Five mutant mice (APP K670 N/M671 L + I716 V + V717I + PS1 M146 L + L286 V) associated with familial AD were selected; that is, 5*∗*FAD mice were selected as experimental animals, half male and half female [5]. In addition, normal mice matched with body weight were selected as the healthy control group and were divided into three groups: healthy control group (*n* = 10), disease group (*n* = 10), and treatment group (*n* = 10, Panax notoginsenoside Rg 1150 mg/kg/d). Panax notoginseng saponin Rg1 is provided by Zhejiang Zuoli Pharmaceutical Group Co., Ltd. Y-maze test was performed before drug treatment, and 5*∗*FAD mice with comparable test scores and healthy control mice were randomly divided into two groups. Because the expression of Abeta in the cortex and hippocampus of 5*∗*FAD mice can begin after 2 months of birth, and cognitive-behavioral abnormalities can occur at 6 months of age, the treatment group began to give a diet mixed with Wuling powder at 4 months of age, and the treatment period was 2 months [6]. The mice in the healthy control group and in the disease group received routine diet.

The rest of this paper is organized as follows.  Section 2 discusses the proposed method.  Section 3 shows the simulation experimental results, and Section 4 concludes the paper with summary and future research directions.

## 2. The Proposed Method

### 2.1. Cognitive Ability Test

The experiment was used to evaluate the spatial learning and memory abilities of animals. The water maze test consists of two parts [7]. The first part tests the learning ability, that is, the positioning navigation test. The pool is divided into four quadrants. The mice are tracked and analyzed automatically from different quadrants every day. If the platform is not found in 120 seconds, the mice are guided to the platform artificially and stay for 20 seconds [8]. The mice were trained for 5 consecutive days, once a day in the morning and afternoon, and the escape latency recorded by the two training centers was regarded as the learning achievement of the mice on the same day on average [9]. The second part carries on the space exploration test. The next day after the achievement test is completed, the platform is removed, and the mice are placed in the same quadrant [10]. The time of mice staying in the quadrant of the platform and the time of crossing the platform within 60 seconds are recorded as indicators of memory.

### 2.2. Y-Shaped Maze Test

The experiment was used to evaluate the learning process that reflected the correct avoidance of passive stimuli in mice. In the experiment, the mice were placed in the starting area to adapt to the environment for 60 seconds, the gate was opened, and then, 36 V AC was introduced. The electric shock button was manipulated to stimulate the mice. The mice would run and escape [11]. For example, the mice escaped to the safety zone in the last run, allowed them to stay in the safety zone for 2 minutes to consolidate their memory, and then removed the mice from the safety zone back to the starting point, repeated electric shocks, repeated training. The correct response was that the mice could enter the safe area directly from the starting point after an electric shock, and the wrong response was that they could enter the safe area through other areas or after scurrying until the mice were successfully trained nine times out of 10 consecutive times [12]. 24 hours later, the number of erroneous reactions in 10 consecutive runs was recorded. The higher the number of erroneous reactions, the lower the ability of learning and memory.

### 2.3. Brain Tissue Detection

After the behavioral test was completed, mice were anesthetized by intraperitoneal injection of 50% sodium pentobarbital (2 ml/kg). PBS and cocktail containing protease inhibitors were perfused into the heart [13]. Half of the brain was preserved in the refrigerator at −80 C for immunoblotting and RT-PCR. The other half was fixed with polyformaldehyde for 24 hours and stored in 30% sucrose/PBS (containing 0.01% sodium azide) for immunohistochemical and immunofluorescence staining.

After the hemispheric tissue was homogenized, the homogenate was divided into three parts. One part was used for immunoblotting assay of APP, CXCR1, Cx43, P2X7, and the other part was used for RT-PCR detection. The first antidilution ratio was 1 : 10,000 anti-APP (22C11), anti-CX3CR1 (1 : 1000), anti-Cx43 (1 : 2000), anti-P2X7 (1 : 300), and antiactin (1 : 500).

Immunohistochemistry and fluorescence staining were performed by ABC method. Frozen sections of tissue are sagittal, 30 μm thick, and all slices concentrated in 0.1 M PH 7.6 phosphate buffer until natural floating [14]. Anti-Abeta 42 (cortical and hippocampal localization, 1 : 2500), anti-Abeta (1 : 500), anti-P2X7 (1 : 200), and anti-Cx43 (1 : 500) were required for immunohistochemistry. After rinsing, biotinylated goat anti-rabbit or goat anti-mouse second antibody (1 : 2000) and ABC complex were added and kept at room temperature for 2 hours, and DAB was colored. Immunofluorescence staining requires the following anti-mice monoclonal antibodies: anti-mouse antibody 4G8 (Abet42, 1 : 10,000 ingested lysosomes), rabbit anti-GFAP (astrocyte, G9269, 1 : 10,000), antineuron-specific nuclear protein (NeuN), rabbit anti-CX3CR1 (1 : 1000), rabbit anti-IBA1 (microglia, 1 : 1000; Sigma), rabbit anti-P2X7 (1 : 300), rabbit anti-Cx43 (1 : 100; Zymed) [15]. After rinsing, the second antibody carrying fluorescent dyes was added, of which Alexa (1 : 1000) was used as fluorescent pigments for A beta 42, thioflavin S, or thiazin red (multiple fluorescent staining for amyloid plaques, neurons, and microglia), Citifluor was used for CX3CR1, and Cy2-conjugated secondary antibody was used for P2X7.

Total RNA of 10 UG was extracted from Trizol solution and then retranscribed to cDNA. Semiquantitative RT-PCR was used to analyze the expression of Cx43 and P2X7. The primers were designed by computer, and the corresponding amplified fragments were enough to cover all target genes [16]. The products were amplified by 2% agarose gel electrophoresis.

### 2.4. Statistical Processing

SPSS 15.0 software was used for statistical analysis, and all data were expressed by *X* + *s*. One-way ANOVA is a method to analyze the results of a single-factor test and test whether a factor has a significant effect on the test results. SNK-q test was used to compare the two groups, and *P* < 0.05 showed significant differences.

## 3. Results

It was found that the escape latency of the treatment group was significantly lower than that of the disease group from the third day of training (*P* < 0.05), indicating that notoginsenoside Rg1 could improve the water maze test results of 5xFAD mice [17].  Table 1 shows water maze test results of 5xFAD mice in different groups.  Figure 1 shows improvement of learning ability in 5*∗*FAD mice.  Figure 2 shows improvement of memory ability in 5*∗*FAD mice.  Table 2 shows the number of erroneous responses of 5xFAD mice to passive stimulation for safe evasion between different groups.

Two months after 150 mg/kg/d treatment, the number of erroneous reactions to passive stimulation to escape safely was significantly lower than that of diseased mice, and the difference was statistically significant. Compared with the healthy control group, there was no statistically significant difference in learning significance between the two groups, although the number of errors after treatment was still higher than that of the control group.  Figure 3 shows the improvement effect of saponin Rg1 on Y-maze test results.

After treatment with notoginsenoside Rg1, the secretion of Cx43 protein in the brain of 5xFAD mice was significantly higher than that of the control group.  Figure 4 shows the secretion of Cx43 protein in the brain.

It was found that the number of reaction errors in the disease group was significantly less than that in the treatment group (*P* < 0.05), indicating that notoginsenoside Rg1 could improve the Y-maze test scores of 5xFAD mice.  Table 2 shows the number of erroneous responses of 5xFAD mice to passive stimulation for safe evasion between different groups.

## 4. Clinical Analysis

The effects of Panax notoginseng saponin Rg1 on cognitive function in 5xFAD mice and the mechanism of Cx43 on improving cognitive function in mice were studied. After treatment with notoginsenoside Rg1, the cognitive ability of 5xFAD mice was significantly improved. At present, the A beta cascade hypothesis is widely accepted as the etiology and exact pathogenesis of AD. In recent years, most of the clinical drugs for AD are these drugs. Panax notoginseng is one of the precious medicinal materials in China. Its alias “Panax notoginseng” and “Tianqi” are mainly distributed in the southwest of China. It belongs to the dried roots and rhizomes of Panax ginseng plants of Acanthopanacis, with sweet, bitter, mild temperature, liver returning, and stomach meridians. Panax notoginseng mainly contains saponins, Panax notoginseng, flavonoid glycosides, volatile oils, amino acids, Panax notoginseng polysaccharides, and a variety of trace elements. It has the functions of stopping bleeding and dissipating blood stasis, detumescence, and pain relief and mainly treats bleeding, swelling, and pain caused by falling. Total saponins of Panax notoginseng are one of the main active components of Panax notoginseng, the content of which is up to 12%. Panax notoginseng saponins are a mixture of more than 20 dammarane saponins. It contains many main active ingredients, such as ginsenoside Rb1, ginsenoside Gg1, and Panax notoginseng saponin Rg1. It plays an important role in blood tonifying, anti-inflammatory, antifatigue, anticancer, and other diseases. It also has the functions of improving memory and cognitive function, inhibiting the damage of amyloid beta-peptide segment, antioxidation, and brain protection. It has the function of treating AD. It has better efficacy. Previous studies have shown that notoginsenoside Rg1 may be involved in the expression of Abeta 42, Cx43, CXCR1, and P2X7, the activation of microglia and astrocytes, and the expression changes of synaptic plasticity markers (PSD-95, synaptic vesicle protein, and p35) in response to cognitive improvement, suggesting that notoginsenoside Rg1 may improve the potential mechanism of pathological damage of Abeta and provide a basis for screening potential clinical drug targets.

Histological study also showed that Cx43 protein expression in the brain of 5xFAD mice was significantly higher than that of the disease group and the normal control group after treatment with notoginsenoside Rg1, which was consistent with the study. Previous studies have found that Panax notoginseng saponin Rg1 improves water maze test scores and promotes hippocampal neurogenesis in rats with depression, and its mechanism is related to the increased expression of Cx43 protein in the brain. Astrocytes, as the most abundant cell type in the brain, are coupled with Cx and play an important role in maintaining the normal function of neuroglial vascular unit. The premise of their role is to maintain a certain level of Cx43 expression; otherwise, they are prone to programmed death. Many studies have confirmed that the overexpression of Cx in astrocytes with periplaque hyperplasia not only weakens the neuroprotective effect, increases the risk of neuronal death [10], but also directly damages neurons.

Another important finding of this study is that the interaction between glia and neurons in 5xFAD mice treated with Panax notoginseng saponin Rg1 is significantly improved. Mei recently observed the temporal and spatial dependence of Cx43 expression in the pathological state of A beta. It was found that the accumulation of A beta activated microglia at the earliest stage, followed by not only an increase in Cx43 expression in astrocytes in the central part of the plaque but also a decrease in Cx43 expression in 15% of astrocytes around the plaque. The increase in Cx43 expression was found to be necessary for astrocyte activation in the study of brain acupuncture injury. Deficiency of CX3CR1 receptor in physiological state may lead to impaired hippocampal-related cognitive function and abnormal neuroplasticity in normal mice. In pathological state, a certain amount of expression is needed, because the removal of CX3CR1 will aggravate the impairment of passive avoidance and novelty exploring behavior, increase the expression of APP, aggravate the pathological damage of tau, and decrease the number of synapses and the calcium binding protein content of hippocampal dentate gyrus neurons. During neuroinflammation, glial cells can transport large amounts of ATP and glutamate to neurons through overexpressed Cx, which leads to neurotoxicity and promotes neuronal death. Increased expression of Cx43 will further promote the release of ATP by astrocytes, and the effect of P2X receptor on microglia will promote the aggravation of inflammation [17]. Therefore, neurons and glial cells interact with each other. The process of action may be a key link in the pathogenesis of AD.

## 5. Conclusion

In order to investigate the effect of notoginsenoside Rg1 on cognitive function in 5*∗*FAD mice and the mechanism of Cx43 in improving cognitive function in mice, the methods 5*∗*FAD mice are selected as experimental animals and normal mice as healthy control. In conclusion, notoginsenoside Rg1 can significantly improve the cognitive function of 5xFAD mice. This study further revealed that notoginsenoside Rg1 plays a role by increasing the secretion of Cx43 protein, thus promoting the reactivity of glial cells and neurons.

## Figures and Tables

**Figure 1:** Improvement of learning ability in 5*∗*FAD mice treated with 137 saponin Rg 1150 mg/kg/d for 2 months can be seen from the graph that the escape latency is significantly reduced compared with the disease group after the third day of training, and the difference is statistically significant (^*∗*^*P* < 0.05, compared with the healthy control group or the treatment group).

**Figure 2:** Improvement of memory ability in 5*∗*FAD mice treated with Rg1-notoginsenoside Rg1150 mg/kg/d for 2 months can be seen from the graph that the duration of stay at the platform quadrant (left) and the number of cross-platform times (right) of the treated mice was significantly increased, and the difference reached statistical significance (^*∗*^*P* < 0.05, compared with the healthy control group or the treatment group).

**Figure 3:** Improvement effect of saponin Rg1 on Y-maze test results shows that the number of false reactions to passive stimulation avoidance in mice treated with 150 mg/kg/d for 2 months was significantly lower than that in diseased mice (^*∗*^*P* < 0.05, compared with the healthy control group or the treatment group). Although the number of errors after treatment was still higher than that in the control group, there was no statistical difference between the two groups.

**Figure 4:** Secretion of Cx43 protein in the brain between the diseased group and the Rg1 treatment group of Panax notoginseng saponin is shown in light red. A1-2 is in the Rg1 treatment group, and B1-2 is in the diseased group (scale bar = 100 um).

**Table 1:** Water maze test results of 5xFAD mice in different groups.

Group	Number of cases (only)	Escape incubation period(s)					Platform image limited residence time	Number of cross-platform trips
		Day1	Day2	Day3	Day4	Day5		
Normal control group	10	120 ± 3.1	103 ± 3.0	98 ± 2.5	70 ± 2.1	58 ± 1.9	45 ± 2.1	6.3 ± 0.8
Disease group	10	120 ± 0.6	98 ± 0.9	63 ± 1.2	43 ± 1.0	38 ± 1.3	19 ± 1.7	1.9 ± 1.2
Treatment group	10	119 ± 1.1	90 ± 1.5	58 ± 1.3	38 ± 1.2	35 ± 1.3	32 ± 1.5	4.6 ± 1.1

**Table 2:** The number of erroneous responses of 5xFAD mice to passive stimulation for safe evasion between different groups.

Group	Number of cases (only)	Number of safe evasion error responses by passive stimulation	
		Before treatment	After treatment

Normal control group	10	2.1 ± 0.9	2.8 ± 0.8
Disease group	10	3.2 ± 1.4	6.3 ± 1.6^*∗*^
Treatment group	10	2.4 ± 0.7	3.9 ± 0.5

## Data Availability

The simulation experiment data used to support the findings of this study are available from the corresponding author upon request.

## References

[1] Ni J., Chen P., Liu Q. (2013). Advance research on strategies for the prevention of Alzheimer’s disease. *Journal of Shenzhen University Science and Engineering*.

[2] Li X., Wang C, Xia Y., Xian S., Pan X. (2016). The relationship between the expression of HMGB1, S100B and RAGE and the occurrence of cognitive dysfunction after cerebral ischemia in rats. *Journal of Wuhan University (Natural Science Edition)*.

[3] Li Z., Li D. (2011). Notoginsenoside Rg1 on learning and memory impairment in rats with post-stroke depression. *PLA Medical Journal*.

[4] Zhang C., Li W., Gu F. (2014). Observation on the efficacy of Panax notoginseng saponin Rg1 in the treatment of post-stroke depression. *Journal of Clinical Neurology*.

[5] Qian Y., Zhan J., Wei D., Zheng Y., Wang X. M., Neurobiology DO (2016). Effects of Shenqi Yizhi Granule on learning and memory ability and content of beta-amyloid protein 1-42 in brain of 5XFAD transgenic mice. *Chinese Journal of Traditional Chinese Medicine Information*.

[6] Koulakoff A., Mei X., Orellana J. A., Sáez J. C., Giaume C. (2012). Glial connexin expression and function in the context of Alzheimer’s disease. *Biochimica et Biophysica Acta (BBA) - Biomembranes*.

[7] Magnotti L. M., Goodenough D. A., Paul D. L. (2011). Deletion of oligodendrocyte Cx32 and astrocyte Cx43 causes white matter vacuolation, astrocyte loss and early mortality. *Glia*.

[8] Chui H. C., Victoroff J. I., Margolin D., Jagust W., Shankle R., Katzman R. (1992). Criteria for the diagnosis of ischemic vascular dementia proposed by the state of California Alzheimer’s disease diagnostic and treatment centers. *Neurology*.

[9] Tang S., Zhang Z., Liu W. (2016). Advances in anti-aging effects of HO-1. *Zhejiang Medical Science*.

[10] Abbasian M, Sayyah M, Babapour V, Mahdian R, Choopani S, Kaviani B (2012). Upregulation of connexins 30 and 32 gap junctions in rat hippocampus at transcription level by chronic central injection of lipopolysaccharide. *Iranian Biomedical Journal*.

[11] Wang L., Li J., Geng M. (2008). Progress in the study of gap junction molecule C x43-related proteins and their functions. *Advances in Modern Biomedicine*.

[12] Mei X., Ezan P., Giaume C., Koulakoff A. (2010). Astroglial connexin immunoreactivity is specifically altered at *β*-amyloid plaques in *β*-amyloid precursor protein/presenilin1 mice. *Neuroscience*.

[13] Theodoric N, Bechberger J. F, Naus C. C, Sin W. C (2012). Role of gap junction protein connexin43 in astrogliosis induced by brain injury. *PLoS One*.

[14] Rogers J. T., Morganti J. M., Bachstetter A. D. (2011). CX3CR1 deficiency leads to impairment of hippocampal cognitive function and synaptic plasticity. *Journal of Neuroscience*.

[15] Jaworski T., Lechat B., Demedts D. (2011). Dendritic degeneration, neurovascular defects, and inflammation precede neuronal loss in a mouse model for tau-mediated neurodegeneration. *American Journal Of Pathology*.

[16] Orellana J. A., Shoji K. F., Abudara V. (2011). Amyloid -induced death in neurons involves glial and neuronal hemichannels. *Journal of Neuroscience*.

[17] Huang C., Han X., Li X. (2012). Critical role of connexin 43 in secondary expansion of traumatic spinal cord injury. *Journal of Neuroscience*.

